# Artificial Intelligence-Based Deep Fusion Model for Pan-Sharpening of Remote Sensing Images

This article has been retracted.

**DOI:** 10.1155/2021/7615106

**Published:** 2021-12-23

**Authors:** Ahmed I. Iskanderani, Ibrahim M. Mehedi, Abdulah Jeza Aljohani, Mohammad Shorfuzzaman, Farzana Akhter, Thangam Palaniswamy, Shaikh Abdul Latif, Abdul Latif, Rahtul Jannat

**Affiliations:** ^1^Department of Electrical and Computer Engineering (ECE), King Abdulaziz University, Jeddah, Saudi Arabia; ^2^Center of Excellence in Intelligence Engineering Systems (CEIES), King Abdulaziz University, Jeddah, Saudi Arabia; ^3^Department of Computer Science, CIT Taif University, Taif, Saudi Arabia; ^4^Aarhus BSS, Aarhus University, Aarhus, Denmark; ^5^Department of Nuclear Engineering, King Abdulaziz University, Jeddah, Saudi Arabia; ^6^Department of Mathematics, King Abdulaziz University, Jeddah, Saudi Arabia; ^7^Department of Electrical and Electronic Engineering (EEE), BRAC University, Dhaka, Bangladesh

## Abstract

During the past two decades, many remote sensing image fusion techniques have been designed to improve the spatial resolution of the low-spatial-resolution multispectral bands. The main objective is fuse the low-resolution multispectral (MS) image and the high-spatial-resolution panchromatic (PAN) image to obtain a fused image having high spatial and spectral information. Recently, many artificial intelligence-based deep learning models have been designed to fuse the remote sensing images. But these models do not consider the inherent image distribution difference between MS and PAN images. Therefore, the obtained fused images may suffer from gradient and color distortion problems. To overcome these problems, in this paper, an efficient artificial intelligence-based deep transfer learning model is proposed. Inception-ResNet-v2 model is improved by using a color-aware perceptual loss (CPL). The obtained fused images are further improved by using gradient channel prior as a postprocessing step. Gradient channel prior is used to preserve the color and gradient information. Extensive experiments are carried out by considering the benchmark datasets. Performance analysis shows that the proposed model can efficiently preserve color and gradient information in the fused remote sensing images than the existing models.

## 1. Introduction

Fusion of multispectral (MS) and panchromatic (PAN) images has attracted researchers' interest, since it results in a fused image with better spatial resolution and spectral information [1]. The spatial resolution of a MS image is significantly better as compared to a PAN image. But a MS image only has a single band. Thus, to obtain an image with significant spectral information and better spatial resolution, efficient pan-sharpening approaches are required [2].

Many pan-sharpening techniques have been implemented so far. The traditional methods suffer from blurring effect and color distortion [1, 3]. Sparse representation theory-based fusion methods can easily overcome the problems of color distortion by enhancing the spatial resolution of MS images [4]. The intensity-hue-saturation (IHS) method was also used to fuse the images. These models were quite simple and efficient and can produce high-spatial-quality images [5, 6]. However, they experience spectral distortion. The spectral fidelity can be enforced using an edge-adaptive IHS method [7]. Compressed sensing (CS) theory is also used for pan-sharpening of multispectral images. It can recover the sparse signal from a small number of linear measurements [8]. Optimized pan-sharpening techniques were also developed to preserve the spectral and geometry constraints [9, 10]. The Bayesian theory-based fusion model solved the problems of linear model and attained superior spatial and spectral fusion [11].

Recently, various deep learning models have been used to implement pan-sharpening techniques to produce HR PAN images. These techniques can effectively model complex relationships between variables via the composition of several levels of non-linearity [12]. In the deep pan-sharpening model, the correlation between the LR/HR MS image patches is the same as the LR/HR PAN image patches. Thereafter, this assumption is used to learn the mapping using convolutional neural network (CNN) [13]. Different types of CNN were used to fuse the images. CNN contains three convolutional layers such input, hidden, and output layers. Activation functions are contained in each layer. Input and hidden layers contain non-linear activation layer while output layer comprises linear activation function. For every layer, there are *I* input bands, *J* output bands, filters, parameters needed to be learned, tensors, weights, and biases. In case of fusion, PAN bands are given as input to the CNN. The components of MS are upsampled and then radiometric indices are extracted. Lastly, non-linear combinations of MS bands are made to improve the performance [14]. However, most of these methods suffer from inadequate spatial texture improvement and spectral distortion issues. To overcome these issues, many techniques were developed. A dual-path fusion network (DPFN) enhanced spatial texture and spectral distortion [15]. Shallow-deep convolutional network (SDCN) can produce fused images with minimal spectral distortion [16]. Dynamic deep learning models were proposed to build sensitive models towards input images [15]. Coupled multiscale convolutional neural network considered the PAN and MS images at different resolutions for better feature extraction [17]. A four-layer CNN and a loss function were designed which can extract spatial and spectral characteristics efficiently from original image. It did not require any refence fused image and hence did not need simulation data for training [18]. Generative adversarial learning (GAN) was also utilized to implement the fusion of PAN and MS images. It has an ability to produce high-fidelity fused images [19].

From the existing literature, it has been found that the deep learning and deep transfer learning models can efficiently fuse the remote sensing images. However, these models do not consider the inherent image distribution difference between MS and PAN images. Therefore, the obtained fused images may suffer from gradient and color distortion problems. To overcome these problems, in this paper, an efficient deep transfer learning model is proposed. The main contributions of this paper are as follows:

1. An efficient Inception-ResNet-v2 model is improved by using a CPL.
2. The obtained fused images are further improved by using gradient channel prior as a postprocessing step.
3. Extensive experiments are carried out by considering the benchmark datasets.

This paper is organized as follows.  Section 2 discusses the literature review.  Section 3 presents the proposed model. Comparative analysis is discussed in Section 4.  Section 5 concludes the paper.

## 2. Literature Review

Wang et al. [20] proposed a pan-sharpening technique based on the channel-spatial attention model (CSA). In this, residual attention module was designed to produce high-resolution images. Xu et al. [21] implemented the soil prediction model using the pan-sharpened remote sensing indices. In this, images of Landsat 8, GeoEye-1, and WorldView-2 were fused. A prediction model was designed using random forest. Ma et al. [22] used the generative adversarial network to implement the pan-sharpening technique. For network training, it did not require ground truth. Akula et al. [23] implemented a pan-sharpening technique using adaptive principal component analysis and local variation contourlet transform. Wang et al. [24] utilized area-to-point regression kriging (ATPRK) for pan-sharpening. Wang et al. [25] presented a pan-sharpening technique based on compressed sensing. The joint sparsity model was used to recover the high-resolution multispectral images.

Wu et al. [26] utilized multiobjective decision for improving the fused multiband images. The information injection model was used to improve texture and gradient details of MS image. Spectral fidelity fusion was designed using injected information and spectral modulation to fused image. Zhuang et al. [27] designed a probabilistic model to fuse MS and PAN images. Gradient domain-guided image filtering was also used to refine the results. The maximum a posteriori model was also implemented on the difference between PAN and MS images and in respective gradient domains too. Sibiya et al. [28] combined image texture obtained from a fused image with partial least squares discriminant analysis to monitor and map commercial forest species. This model proved that the image texture can discriminate commercial forest species.

Fang et al. [29] designed a framelet-based fusion model by using a variational model. The split Bregman iteration was also used to obtain better results. The Bregman method solves the convex optimization problems using regularization. It is best suited for those optimization problems where constraints are well specified. Due to error cancellation effect, it converges very fast. Wang et al. [30] proposed sparse tensor neighbor embedding for fusion of PAN and MS images using N-way block pursuit. A sparse tensor was concatenated with neighbor embedding to obtain a new high-dimensional sparse tensor embedding for fusion of PAN and MS images in an efficient manner. Saeedi and Faez [31] utilized shiftable contourlet transform and multiobjective particle swarm optimization (MPSO) to fuse PAN and MS images. PAN and MS images were histogram matched prior to fusion process. Fang et al. [32] designed a pan-sharpening technique using variational approach. In this, three assumptions were made to construct the energy function. The minimized solution was obtained using the Bregman algorithm. Zhang et al. [33] implemented a variational energy function to preserve the spectrum, geometry, and correlation information of the original images while pan-sharpening.

Ye et al. [34] proposed gradient-based deep network prior to fuse PAN and MS images. Convolutional neural network (CNN) was trained in gradient domain using the problem-specific recursive block. Xing et al. [35] implemented the pan-sharpening technique using deep metric learning (DML). The deep metric learning was used to train refined geometric multimanifold neighbor embedding. The hierarchical characteristics of masks were used by considering various non-linear deep learning models. Gogineni and Chaturvedi [36] used multiscale learned dictionary (MSLD) to design a pan-sharpening technique. It could obtain the underlying features of images, in which the characteristics of both learned dictionaries and multiscale were possessed. Huang et al. [37] developed a fusion model using multiple deep learning models (MDLMs). The non-subsampled contourlet transform (NSCT) used to decompose the PAN images into frequency bands. The characteristics of high-frequency bands were learned by the deep learning model.

From the literature, it is found that the deep learning model should be improved by using a better loss function and some preprocessing techniques [38–40].

## 3. Proposed Model

An efficient artificial intelligence-based deep transfer learning model is proposed. Inception-ResNet-v2 model is improved by using a CPL. The obtained fused images are further improved by using gradient channel prior as a postprocessing step.

### 3.1. Inception-ResNet-v2

Inception-ResNet-v2 is a well-known model which is improved InceptionNet with residual connections. It is achieved by replacing the filter concatenation stage of the InceptionNet (see [41]).  Figure 1 shows the architecture of Inception-ResNet-v2.

### 3.2. Color-Aware Perceptual Loss

CPL [42] is utilized to assign small coefficients to feature channels which are more sensitive to colors for every *L* Inception-ResNet-v2 layer during the computation of perceptual loss.

The difference among the respective color and a grayscale-inverted MS image (*M*_*δ*_^−1^) is utilized to compute coefficients of features. Higher difference indicates that the features are more sensitive to colors. CPL is also more sensitive to gradient information. The average feature difference is then assigned to the exponential function with a variable *γ* (see [42]). It can be represented as

(1) $$\begin{array}{c} M_{\delta }^{-1}=1-\frac{\left(M_{\gamma }^{R}+M_{\gamma }^{G}+M_{\gamma }^{B}\right)}{3}, \end{array}$$

where *M*_*γ*_^*R*^, *M*_*γ*_^*G*^, and *M*_*γ*_^*B*^ represent color channels of MS image. The CPL coefficients for color channels of every layer *l*, **W**_*cpl*_^*l*^, can be computed as

(2) $$\begin{array}{c} W_{cpl}^{l}=e^{-\gamma \left(1/N\right)\sum_{n}^{N}\left|\phi^{l}\left(M_{\delta }^{-1}\right)-\phi^{l}\left(M_{\gamma }\right)\right|}, \end{array}$$

where *γ* is used to neglect features which are sensitive to colors. For PAN image (*M*_*pc*_) and a CNN-based fused image (*M*_*ps*_), CPL can be computed as

(3) $$\begin{array}{c} l_{cpl}={\sum_{l=1}^{L}\left\|W_{cpl}^{l}⊙\left(\phi_{m_{l}}^{l}\left(M_{pc}\right)-\phi_{m_{l}}^{l}\left(M_{ps}\right)\right)\right\|}_{1}, \end{array}$$

where *m*_*l*_=[7,5,3] shows the size of max-pool implemented on *l*^th^ layer feature which is used to achieve average of shift invariance to CPL. It can efficiently manage the misalignment problem.

Although CPL assigns high-frequency information to *M*_*ps*_, additional loss is also required for color fidelity. Therefore, the perceptual and *l*_1_ losses are used. The fidelity loss can be defined as

(4) $$\begin{array}{c} l_{f}=\alpha_{cpl}l_{cpl}\left(M_{pc},M_{ps}\right)+\alpha_{\gamma }l_{p}\left(M_{\gamma },M_{ps↓}\right)+\alpha_{l1}l_{1}\left(M_{\gamma },M_{ps↓}\right), \end{array}$$

where *M*_*ps*↓_ shows a downscaled PS image to the MS resolution, *l*_1_ loss is an average absolute difference, i.e., 1/*N*∑_*n*_^*N*^|*M*_*γ*_ − *M*_*ps*↓_|, and *α*_*cpl*_, *α*_*γ*_, and *α*_*l*1_ are set to 0.85, 0.02, and 0.95, respectively.

### 3.3. Gradient Channel Prior

GCP is utilized to restore any kind of degradation from the images. It has an ability to preserve the gradient and texture information of restored images [43]. GCP can be defined as

(5) $$\begin{array}{c} \nabla I\left(m,n\right)=\left(\begin{array}{c} \psi_{m}\\ \psi_{n} \end{array}\right)=\left(\begin{array}{c} \partial I/\partial m\\ \partial I/\partial n \end{array}\right). \end{array}$$

An amplitude of *I* can be computed as

(6) $$\begin{array}{c} \text{mag}\left(I\right)=\sqrt{\left(\psi_{m}^{2}+\psi_{n}^{2}\right)}. \end{array}$$

An orientation angle of ∇*I* can be computed as

(7) $$\begin{array}{c} \nabla_{O}\left(m,n\right)=\text{arctan}\left(\frac{\psi_{n}}{\psi_{m}}\right). \end{array}$$

For *I*(*m*, *n*), *ψ*_*m*_ and *ψ*_*n*_ can be computed using various masks (see [44]).

## 4. Performance Analysis

The proposed model is trained on using 100 epochs with a mini-batch size of 10 using Adam optimizer [45]. The learning rate is used as 5 × 10^−5^. All experiments are performed on MATLAB2021a software. Experiments are performed on Pleiades, QuickBird, IKONOS, and WorldView-2 images. Comparisons are performed with six well-known competitive techniques.

### 4.1. Visual Analysis

Figures 2 and 3 show the visual analysis of the proposed model. It is found that the proposed model has better visibility as compared to the existing techniques. Red rectangles show the specific region in the obtained fused images. The selected region reflects the spatial and spectral information along with any kind of artifacts which are present in the obtained fused images. Also, the proposed model shows better gradient and color preservation as compared to the existing techniques. The results obtained from the proposed model show better spatial and spectral information. It clearly shows that the existing models are able to fuse the images by improving the spatial and spectral information of fused images. But whenever there is redundant information in both PAN and MS images, then the existing method fails to fuse the content efficiently. Also, the texture and gradient preservation is significantly more in the fused image obtained using the proposed model.

### 4.2. Quantitative Analysis

Five well-known quality metrics, i.e., root mean square error (RMSE) [46], universal image quality index (UIQI) [47], correlation coefficient (CC) [46], spectral angle mapper (SAM) [46], and Erreur relative globale adimensionnelle de synthese (ERGAS) [48], are used for comparative analysis.

Table 1 shows CC analysis of the proposed deep pan-sharpening model. CC is desirable to be maximum. It is found that the proposed model outperforms the competitive pan-sharpening models by 1.7824%.

Table 2 depicts UIQI analysis of the proposed deep pan-sharpening model. UIQI is desirable to be maximum. It is found that the proposed model outperforms the competitive pan-sharpening models by 1.2498%.

Table 3 shows SAM analysis of the proposed deep pan-sharpening model. SAM is desirable to be minimum. It is found that the proposed model outperforms the competitive pan-sharpening models by showing an average reduction of 1.3457%.

The quality of pan-sharpened images can be assessed using ERGAS. It determines the transition between spectral and spatial information [49].  Table 4 demonstrates ERGAS analysis of the proposed deep pan-sharpening model. ERGAS is desirable to be minimum. It is found that the proposed model outperforms the competitive pan-sharpening models by showing an average reduction of 1.0985%.

Table 5 demonstrates RMSE analysis of the proposed deep pan-sharpening model. RMSE is desirable to be minimum. It is found that the proposed model outperforms the competitive pan-sharpening models by showing an average reduction of 1.5486%.

## 5. Conclusion

To obtain a remote sensing image with better spatial and spectral information, efficient image fusion techniques are desirable. However, it has been found that the existing models do not consider the inherent image distribution difference between MS and PAN images. Therefore, the obtained fused images suffer from gradient and color distortion problems. To overcome these problems, in this paper, an efficient deep transfer learning model has been proposed. Inception-ResNet-v2 model was improved by using a color-aware perceptual loss (CPL). The obtained fused images were further improved by using gradient channel prior as a postprocessing step. Gradient channel prior was utilized to preserve the color and gradient information. Extensive experiments were carried out by considering the benchmark datasets. Performance analysis has shown that the proposed model can efficiently preserve color and gradient information in the fused remote sensing images than the existing models. The proposed model outperformed the competitive pan-sharpening models in terms of CC and UIQI by 1.7824% and 1.2498%, respectively. Also, compared to the existing models, the proposed model has achieved an average reduction in SAM, ERGAS, and RMSE by 1.3457%, 1.2847%, and 1.5486%, respectively.

## Figures and Tables

**Figure 1:** Architecture of Inception-ResNet-v2.

**Figure 2:** Visual analysis of pan-sharpening techniques. (a) Low-resolution multispectral (MS) image. (b) High-spatial-resolution panchromatic (PAN) image.

**Figure 3:** Visual analysis of pan-sharpening techniques. (a) Low-resolution multispectral (MS) image. (b) High-spatial-resolution panchromatic (PAN) image.

**Table 1:** Analysis of correlation coefficient (maximum is desirable).

Images	CSA	CNN	MSLD	MDLM	DML	MPSO	Proposed
Pleiades 1	0.9482	0.9585	0.9525	0.9356	0.9495	0.9531	**0.9612**
Pleiades 2	0.9384	0.9545	0.9588	0.9636	0.9595	0.9594	**0.9668**
QuickBird 1	0.9543	0.9525	0.9517	0.9594	0.9353	0.9406	**0.9626**
QuickBird 2	0.9388	0.9387	0.9627	0.9435	0.9451	0.9388	**0.9659**
QuickBird 3	0.9422	0.9451	0.9386	0.9457	0.9481	0.9416	**0.9513**
IKONOS 1	0.9601	0.9493	0.9589	0.9366	0.9547	0.9645	**0.9677**
IKONOS 2	0.9391	0.9617	0.9442	0.9452	0.9405	0.9578	**0.9649**
IKONOS 3	0.9422	0.9562	0.9385	0.9563	0.9602	0.9529	**0.9634**
WorldView-2 1	0.9399	0.9572	0.9609	0.9533	0.9401	0.9549	**0.9641**
WorldView-2 2	0.9446	0.9418	0.9393	0.9386	0.9528	0.9537	**0.9569**

**Table 2:** Analysis of UIQI (maximum is desirable).

Images	CSA	CNN	MSLD	MDLM	DML	MPSO	Proposed
Pleiades 1	0.8227	0.8253	0.8252	0.8256	0.8207	0.8163	**0.8288**
Pleiades 2	0.8286	0.8222	0.8168	0.8277	0.8333	0.8303	**0.8365**
QuickBird 1	0.8276	0.8292	0.8161	0.8247	0.8219	0.8238	**0.8324**
QuickBird 2	0.8324	0.8235	0.8182	0.8235	0.8188	0.8276	**0.8356**
QuickBird 3	0.8176	0.8302	0.8216	0.8310	0.8322	0.8157	**0.8354**
IKONOS 1	0.8253	0.8205	0.8152	0.8266	0.8155	0.8253	**0.8298**
IKONOS 2	0.8324	0.8335	0.8325	0.8337	0.8305	0.8254	**0.8369**
IKONOS 3	0.8209	0.8338	0.8292	0.8154	0.8249	0.8237	**0.8375**
WorldView-2 1	0.8236	0.8347	0.8165	0.8294	0.8304	0.8253	**0.8379**
WorldView-2 2	0.8185	0.8183	0.8275	0.8236	0.8216	0.8323	**0.8355**

**Table 3:** Analysis of SAM (minimum is desirable).

Images	CSA	CNN	MSLD	MDLM	DML	MPSO	Proposed
Pleiades 1	6.1233	5.2497	4.8504	5.2314	5.6140	5.7876	**4.8472**
Pleiades 2	5.0322	5.0038	5.2320	5.6089	5.0142	5.027	**5.0006**
QuickBird 1	5.5875	5.7493	5.6528	5.5909	5.5925	5.1086	**5.1054**
QuickBird 2	5.3167	4.9801	5.2275	5.4522	5.0770	4.8495	**4.8463**
QuickBird 3	4.8664	5.4697	5.5565	5.4524	5.6393	4.9815	**4.8632**
IKONOS 1	5.6374	4.9882	4.8493	5.3591	4.9381	5.4698	**4.8461**
IKONOS 2	5.5923	5.4901	5.5478	4.8991	5.7502	5.7276	**4.8959**
IKONOS 3	5.1743	4.8863	5.6782	5.0255	5.1709	5.0138	**4.8831**
WorldView-2 1	5.4105	5.1662	5.6827	5.6985	5.8012	5.3316	**5.1635**
WorldView-2 2	5.0545	4.8830	5.3821	5.3335	5.0876	5.5423	**4.8798**

**Table 4:** Analysis of ERGAS (minimum is desirable).

Images	CSA	CNN	MSLD	MDLM	DML	MPSO	Proposed
Pleiades 1	6.4651	5.7022	6.0366	5.5356	7.0193	6.5008	**3.0324**
Pleiades 2	7.0733	6.7986	5.5258	5.8420	7.5852	7.1921	**3.7944**
QuickBird 1	5.1640	6.2983	7.1174	5.6054	7.0157	5.8708	**3.2941**
QuickBird 2	6.2149	6.3734	7.7259	7.4269	6.0897	6.6930	**3.0855**
QuickBird 3	5.3291	6.4481	6.4994	7.0956	6.7466	6.5206	**3.4439**
IKONOS 1	5.0443	7.5506	5.3478	5.6993	7.6662	7.9703	**2.9661**
IKONOS 2	5.4928	7.2282	6.8215	6.2475	5.4354	5.0493	**3.2433**
IKONOS 3	7.3333	5.2985	5.9716	7.3313	6.4497	6.4498	**3.4455**
WorldView-2 1	7.3629	5.9718	7.6287	6.0475	7.1961	5.4670	**4.0428**
WorldView-2 2	5.9306	6.9576	6.2451	6.6974	7.1292	5.8911	**3.2409**

**Table 5:** Analysis of RMSE (minimum is desirable).

Images	CSA	CNN	MSLD	MDLM	DML	MPSO	Proposed
Pleiades 1	17.3301	17.5812	17.0435	18.6407	17.5075	18.8094	**16.9898**
Pleiades 2	17.4840	17.4399	17.883	18.6324	17.2132	17.7383	**17.1600**
QuickBird 1	16.9437	17.2044	17.3443	18.1278	18.4979	18.7183	**16.8905**
QuickBird 2	18.7044	17.9968	17.2075	18.698	18.3412	18.3956	**17.1543**
QuickBird 3	18.2260	18.7599	17.5858	16.9439	16.9921	18.1098	**16.8907**
IKONOS 1	18.7411	17.6879	17.9462	17.4335	17.9966	17.1842	**17.1314**
IKONOS 2	17.9322	18.275	18.2602	18.1607	17.2863	16.9537	**16.9005**
IKONOS 3	17.0796	17.8841	18.5387	17.9606	17.7461	17.8408	**17.0264**
WorldView-2 1	17.9519	17.5074	17.3929	18.5105	18.4653	17.1286	**17.0754**
WorldView-2 2	17.0827	18.5631	17.5701	18.6942	17.1731	18.1685	**17.0295**

## Data Availability

The data used to support the findings of this study are included within the article.
